# Exploring Occupational Health Challenges in Pathology: A Cross-Sectional Survey of Indian Pathologists

This article has been retracted.

**DOI:** 10.7759/cureus.75264

**Published:** 2024-12-07

**Authors:** Rahul Kanungo, Anjali Sharma, Sajal Pagi, Kanika Sachar

**Affiliations:** 1 Pathology, BLDE (Deemed to be University) Shri B.M. Patil Medical College, Hospital, and Research Centre, Vijayapura, IND

**Keywords:** cut injury, ergonomics, formalin, musculoskeletal, needlestick injury, occupational hazards, pathologist, safety practices

## Abstract

Introduction

Occupational health hazards are a significant concern for pathologists due to their unique work environment. These professionals face risks from prolonged microscope use, exposure to chemicals such as formalin, and handling sharp instruments, leading to issues such as musculoskeletal disorders and needlestick injuries. Addressing these hazards is crucial for their well-being and the overall efficiency of medical diagnostics. Implementing effective safety measures and increasing awareness can create a safer and healthier workplace for pathologists.

Objective

This study primarily aimed to assess the prevalence of occupational health hazards among Indian pathologists. It further assessed the knowledge and attitudes of pathologists toward safety practices in pathology. Specifically, it explored the research questions: What are the levels of awareness and adherence to safe practices among pathologists? What common factors contribute to reluctance in following these practices, particularly concerning occupational hazards such as musculoskeletal disorders, cut injuries, and chemical exposure?

Materials and methods

Online and offline versions of a survey questionnaire were prepared to cover the spectrum of occupational hazards regarding musculoskeletal diseases, cut injuries, and level of awareness. The questionnaire was shared through email and social networking platforms with over 1000 pathologists across India. The responses, inputs, and open-ended comments from the respondents were collected and analyzed.

Results

A total of 146 pathologists responded and completed the survey, starting from residents to professors. Almost all of them had experienced musculoskeletal problems, among which neck pain was the predominant problem, accounting for 82 (56.2%), followed by low back aches, accounting for 69 (47.3%). Needlestick injury was reported by 33 (22.6%) as “at least once in the past year.” Cut-related injury while performing grossing/autopsy was reported by 57 (39%), and 29 (19.8%) pathologists sustained this cut-related injury once within the last one year. A total of 26 (17.8%) pathologists had been injured two to five times, and two pathologists (1.3%) had this injury more than five times within last one year. Over half of the respondents, i.e., 90 (61.6%) pathologists, reported eye fatigue symptoms. Additionally, 94 (64.3%) pathologists reported an increase in refractive error after joining the practice, with myopia being the most common, affecting 69 (47.2%) pathologists. Adverse reactions to formalin were reported by 96 (66%) of the 146 respondents. These findings highlight the need for ergonomic interventions and stricter safety protocols in pathology laboratories.

Conclusion

The study highlights substantial occupational health challenges among Indian pathologists, particularly musculoskeletal issues, needlestick and cut injuries, eye strain, and adverse effects of formalin exposure. These findings emphasize the urgent need for enhanced safety training and compliance with best practices to mitigate health risks, improve occupational well-being, and support the sustainability of pathology practice in India.

## Introduction

Pathologists play a critical role in the healthcare system, operating within environments that expose them to a variety of occupational health risks. Globally, occupational health issues in pathology are an increasing concern due to prolonged periods of microscope and computer use, necessitating constant sitting, often in ergonomically challenging positions [1]. This sedentary work setup predisposes pathologists to musculoskeletal disorders, while their exposure to infectious materials (e.g., blood and tissue samples) raises the risk of transmission-related injuries, such as needlestick injuries, during procedures such as fine needle aspiration cytology [1-3]. As healthcare demands grow worldwide, the burden of these occupational health challenges for pathologists intensifies, impacting not only their personal well-being but also the efficacy of diagnostic services.

In addition to the aforementioned occupational challenges, pathologists routinely encounter formalin, a ubiquitous chemical widely employed in pathology laboratories. Despite its integral role in pathology practices, prolonged exposure to formalin is known to pose health risks. The chemical has been associated with various harmful effects, ranging from respiratory and skin irritation to more severe concerns such as its potential carcinogenic properties [4,5].

A well-established understanding of occupational health issues within the field of pathology makes the case for having a plan to prevent the possibility of injuries. Hence, it is essential to understand the gap between theoretical knowledge and the practical implementation of safety measures. In many cases, safety measures are cheaper and very effective, such as using cut-resistant gloves to prevent cut-related injuries [6-8].

Even though the knowledge about the safe practices to be followed is high among healthcare professionals, there is very little data available on the occupational health hazards among pathologists in India. This article seeks to delve into the knowledge, attitudes, and practices regarding occupational health among pathologists, considering distinct professional categories such as residents, professors, and private practitioners. By shedding light on these aspects, we aim to identify areas where safety protocols can be bolstered. Beyond a mere assessment, this study aspires to function as a sensitization tool, fostering a deeper appreciation for occupational hazards among pathologists. The findings are expected to stimulate further exploration in the field and contribute to the development of tailored guidelines for the prevention of musculoskeletal disorders, needle-related injuries, cuts, and exposure to infectious and carcinogenic agents, with a specific focus on the unique challenges posed by the Indian work environment.

Objectives of the study

This study sought to explore the prevalence of occupational health hazards among pathologists in India and identify common factors contributing to reluctance in adhering to safe procedures, focusing on occupational hazards related to musculoskeletal diseases, cut injuries, and overall awareness within the pathology community. It further aimed to assess the knowledge and attitudes of pathologists toward safety practices in pathology.

## Materials and methods

Study design

The present study was a descriptive cross-sectional study aimed at assessing the occupational hazards faced by pathologists in India over a period of six months, from June 2022 to December 2022. The study was conducted over three phases, targeting pathologists working in various institutions across the country. Data were collected through a structured questionnaire distributed both online and in printed form.

Study population

The study population consisted of pathologists at different stages of their careers, including residents, professors, and practicing pathologists. A total of 1,000 pathologists across India were approached to participate in the survey, out of which 146 completed the questionnaire. The participants included pathologists from government institutions, non-government institutions, corporate hospitals, and private practice settings, ensuring a wide representation of the pathology community.

Inclusion and exclusion criteria

The study included all pathologists registered with the Karnataka Chapter of the Indian Association of Pathologists and Microbiologists (KCIAPM) and the Indian Association of Pathologists and Microbiologists (IAPM), working at all types of institutions, including government, private, and corporate hospitals. Participants were selected if they had at least one year of experience in pathology. Those who did not consent to participate or failed to complete the questionnaire within the date of expiry (August 2022) were excluded from the study.

Study procedure

The study was conducted in three phases. Phase I involved collecting data from pathologists within the Department of Pathology at BLDE (Deemed to be University), Shri B.M. Patil Medical College, Hospital, and Research Centre, Vijayapura. Phase II extended the survey to pathologists registered under the KCIAPM. In phase III (final phase), the survey was distributed nationwide to members of the IAPM. The questionnaire was distributed via email, and responses were collected both through email and printed forms where necessary. Follow-up emails were sent 15 days after the initial request to maximize participation.

Data collection tool

A structured questionnaire was developed by the authors (included in Appendices). The questionnaire aimed to capture data on the knowledge, attitudes, and practices regarding occupational hazards, focusing on areas such as musculoskeletal disorders (neck pain, back pain, eye strain), chemical hazards (exposure to formalin, xylene), procedural risks (needlestick and cut-related injuries during grossing/autopsy). The questionnaire also included demographic details, professional experience, working hours, and institutional affiliation. Open-ended questions allowed participants to provide additional insights or suggestions. Pilot testing of the questionnaire was performed using 13 pathologists from the institute's Department of Pathology.

Data collection and distribution

The questionnaire was distributed via two methods. The first method was an online survey, carried out with the help of a Google Form (Google LLC, Mountain View, California, United States). A Google Form link was shared via email and social networking platforms (WhatsApp [Meta Platforms, Inc., Menlo Park, California, United States] groups) to over 1,000 pathologists. To ensure broad coverage and avoid duplication of responses, each participant's email address was used as a unique identifier, and limits were set to a maximum of one response per user. Reminders and follow-up emails were sent to enhance response rates.

The second method was an offline survey carried out with the help of printed version of the same Google Form, circulated to pathologists at various pathology conferences.

Statistical analysis

Chi-square and Fisher-exact tests were used as tests of association between the different variables. The incidences of musculoskeletal diseases, needlestick injury, and chronic diseases were calculated by dividing the total number of new cases under each category over the study period by the baseline population. Statistical analysis was conducted using SPSS, Version 20.0 (IBM Corp., Armonk, NY). A p-value less than 0.05 was considered statistically significant.

Ethical considerations

The study protocol was approved by the Institutional Ethics Committee of BLDE (Deemed to be University), Shri B.M. Patil Medical College, Hospital, and Research Centre on 21 April 2022 as per approval number BLDE(DU)/IEC/401/22-23. Participation was voluntary, and informed consent was obtained from all respondents before completing the survey. Confidentiality of the participants' data was maintained throughout the study.

## Results

The online questionnaire was completed by 146 doctors out of over 1,000 pathologists who were contacted through email, social networking groups, and printed questionnaires at conferences. The mean age of respondents was 34 years, with a standard deviation of 9.5 years (34.0±9.5). The youngest participant was 25 years old, and the oldest was 67 years old (Figure 1).

**Figure 1:** Distribution of respondents according to age groups.

The majority of respondents were female, accounting for 88 (60.3%) of the total 146 respondents, and males accounted for 58 (39.7%) of the total (Figure 2).

**Figure 2:** Distribution of respondents according to gender.

The majority of respondents were postgraduates, making up 76 (52.1%) of the total 146 samples. This was followed by consultant pathologists with more than 15 years of experience, accounting for 27 responses (18.5%). Next, 24 respondents (16.4%) had three to eight years of experience, and 19 respondents (13%) had eight to 15 years of experience (Figure 3).

**Figure 3:** Distribution of respondents according to different levels of experience at workplace.

Most respondents, i.e., 76 (52.1%) worked in non-government institutions, followed by 43 (29.5%) in government institutions, 11 (7.5%) in corporate hospitals, and 11 (7.5%) pursuing private practice (Figure 4).

**Figure 4:** Distribution of respondents according to nature of workplace.

About 44.5% of respondents (N=65) had mean weekly working hours more than 50 per week, whereas the rest worked less than or equal to 50 hours per week (Figure 5).

**Figure 5:** Distribution of respondents according to number of work hours per week.

When asked about the reporting of injuries at workplace, 43.2% (N=63) replied with a yes, 41.1% (N=60) with a no due to the absence of a reporting protocol, and 15.8% (N=23) again with a no because of a lack of awareness (Figure 6).

**Figure 6:** Responses of different participants regarding reporting of injuries at workplace.

When asked to specify the reason for not using ergonomically designed microscopes, 59.2% (N=86) were not aware of them, 34.2% (N=50) stated they were too expensive, and 6.6% (N=10) were using them but found that they did not prevent musculoskeletal problems.

Musculoskeletal disorders

About 56.2% (N=82) of respondents suffered from neck pain, followed by 47.3% (N=69) who suffered from low backache. One respondent (0.7%) suffered from shoulder pain. Additionally, 61.6% (N=90) reported symptoms of eye fatigue, and 55.4% (N=81) reported an increase in refractive error after joining the practice, with the predominant refractive error being myopia in 47.2% of the respondents (N=69) (Figure 7).

**Figure 7:** Prevalence of the different types of musculoskeletal injuries faced by the participants.

Therefore, neck pain and low back ache among majority of respondents highlight the importance of proper posture while sitting for long reporting hours.

Needlestick injury

Out of 146 respondents, 50 (34.2%) experienced a needlestick injury in the past year. Of these, 33 (66%) had a needlestick injury once in the last year, 16 (32%) had it one to five times in the last year, and only 1 (2%) had it more than five times (Figure 8).

**Figure 8:** Incidence of needlestick injury among the respondents.

Needlestick injuries were most prevalent among younger professionals, indicating a need for targeted safety training.

Cut-related injury

Cut-related injury while performing grossing/autopsy was reported by 57 (39%) respondents. Of these, 29 (50.8%) respondents sustained this cut-related injury once in the last one year, 26 (45.6%) sustained it two to five times, and 2 (3.6%) sustained it for more than five times in last one year (Figure 9).

**Figure 9:** Prevalence of cut-related injury among the respondents.

Cut-related injuries were prevalent among almost 40% (N=58) of professionals, with majority of them facing it once in a year. 

Other chronic conditions

The number of respondents suffering from chronic diseases was found to be 37% (N=54) of the total number of respondents (N=146). Among these, the predominant chronic conditions reported were hypertension, i.e., 40.7% (N=22), followed by diabetes, i.e., 27.7% (N=15). This was followed by burnout, which was reported by 22.2% (N=12) of respondents, and cervical disc prolapse by 13% (N=7) of respondents. Other chronic conditions noted in lesser number of respondents included depression, tuberculosis, and contact dermatitis. Depression was found affecting 9.2% (N=5) of respondents, followed by tuberculosis in 3.7% (N=2), and contact dermatitis in 1.8% (N=1) of the total number of respondents who reported having suffered from at least one of the above chronic conditions (Figure 10).

**Figure 10:** Prevalence of different types of chronic conditions within the participants.

Therefore, among those participants who suffered chronic conditions, majority suffered from hypertension, followed by diabetes and burnout.

Adverse reactions to formalin exposure

Around 66% (N=96) of the total 146 respondents admitted to having adverse reactions to formalin exposure, highlighting the urgent need for stringent measures regarding its exposure reduction (Figure 11).

**Figure 11:** Prevalence of adverse reactions to formalin exposure among the respondents.

Incidences of musculoskeletal diseases, needlestick injury, and chronic conditions

Our study revealed a high prevalence of musculoskeletal issues among pathologists, with neck pain (34.7%, N=50) and low back ache (25.2%, N=37) being the most common, emphasizing the need for ergonomic interventions. Chronic diseases were reported by 44.9% (N=65) of participants, with mental health concerns such as depression (12.9%, N=19) and burnout (9.5%, N=14) being significant, highlighting the importance of mental well-being initiatives at the workplace. Additionally, 37% (N=54) of respondents reported experiencing needlestick injuries, underlining the urgent requirement for strict safety protocols and protective measures in pathology laboratories. The summary of these incidences has been provided in Table 1 below.

**Table 1:** Incidence of musculoskeletal diseases, chronic conditions, and needlestick injuries among the respondents.

Hazard Type	Category	Incidence (%)
Musculoskeletal Diseases	Neck Pain	34.7%
	Low Back Ache	25.2%
	Both Neck and Low Back Ache	21.1%
	No Issues Reported	15.0%
	Others	~0.7%
Chronic Diseases	No Chronic Diseases	55.1%
	Depression	12.9%
	Burnout	9.5%
	Combined Conditions (e.g., Burnout and Depression)	~5.4%
	Less Frequent (Hypertension, Diabetes, Tuberculosis)	<4%
Needlestick Injuries	No Incidents	63.0%
	One Incident	24.4%
	1-5 Incidents	11.9%
	>5 Incidents	0.7%

Our study revealed both significant and non-significant findings related to occupational hazards among pathologists. Musculoskeletal problems were highly prevalent, with neck pain (34.7%, N=50) and low back ache (25.2%, N=37) being the most common; however, no significant association was found between gender and musculoskeletal issues (p=0.353). Similarly, the use of ergonomic chairs showed no significant association with gender (p=0.240), indicating that other factors, such as workplace policies, may play a larger role. A significant association was observed between workplace type and the use of ergonomic microscopes (p=0.004), highlighting disparities in ergonomic tool accessibility. Needlestick injuries were reported by 54 (37%) participants, but the association between workplace type and these injuries was not significant (p=0.218). These findings emphasize the need for universal ergonomic interventions and safety protocols while addressing systemic barriers to access and implementation.

## Discussion

Occupational hazards in pathology are an enduring concern, and various studies have sought to explore these challenges in different contexts. Our study sheds light on the occupational health issues faced by pathologists in India, with particular emphasis on musculoskeletal disorders, chemical hazards such as formalin exposure, and procedural risks such as needlestick and cut-related injuries. By comparing our findings with previous studies, we can better understand the global relevance and specificity of these occupational hazards within Indian pathology practice.

In line with our study, which found that 56.2% (N=82) of respondents reported neck pain and 47.3% (N=69) experienced low back pain, Richtsmeier et al. also highlighted musculoskeletal disorders as a major concern for pathologists [9]. Richtsmeier’s study emphasized the use of ergonomic chairs and microscopes as effective preventative measures​. Although awareness about ergonomic interventions is relatively high, as shown in previous literature, the actual use of ergonomically designed microscopes and chairs is limited due to high costs and lack of availability in many institutions. This gap was also noted by Fritzsche et al., who emphasized the need for greater accessibility to these tools [10]​. Institutional investment in ergonomic equipment could help solve these issues [11]. In another study by Fritzsche et al., it was noted that knowledge about these tools is high, but their use is limited, particularly due to cost and availability​ [12]. Our study echoes this sentiment, with many respondents citing the high cost and inaccessibility of ergonomic equipment as barriers to its use. To bridge this gap, hospitals and pathology labs in India need to prioritize occupational health and invest in affordable ergonomic solutions that can enhance the well-being and productivity of their workforce [13].

The health risks posed by formaldehyde are well-documented, and our study found that 66% (N=96) of pathologists reported formalin intolerance. This is consistent with studies by the International Agency for Research on Cancer (IARC) and the National Toxicology Program (NTP), which have linked formaldehyde exposure to nasopharyngeal carcinoma and leukemia​ [14]. Similarly, pathologists and residents, particularly during sample grossing, experienced notable formaldehyde exposure with levels surpassing the occupational exposure limit according to a study conducted by Silvia Fustinoni et al. [15]. Despite the availability of guidelines, our study shows that many Indian laboratories lack proper protective measures and ventilation systems to ensure safe levels of formaldehyde exposure [15]. Fritzsche et al. also pointed out that the protective measures available are not used to their full potential in many labs [10]​. In contrast to countries with more stringent regulatory oversight, where formaldehyde substitutes or better ventilation systems are commonplace, Indian pathology labs often operate with minimal safety protocols due to financial constraints and institutional neglect. This highlights a crucial area where improvements can be made to safeguard the health of pathologists.

Our study revealed that 34.2% (N=50) of pathologists experienced needlestick injuries, and 39% (N=57) reported cut-related injuries during grossing or autopsy. These findings align with Fritzsche et al., who found that needlestick and cut-related injuries are significant occupational hazards in pathology [12]​. Both studies agree that the knowledge of preventive measures, such as using cut-resistant gloves, is high, but actual practice lags behind. The reasons for not using protective gear, such as cut-resistant gloves, include discomfort, loss of dexterity, and overconfidence in one’s technique. Richtsmeier et al. also emphasized the effectiveness and cost-efficiency of cut-resistant gloves in preventing such injuries [9]​. However, in the Indian context, as demonstrated by our study, financial barriers and institutional negligence further hinder the adoption of these safety measures. In contrast, studies conducted in more developed healthcare settings report higher adherence to safety protocols due to better resource availability and regulatory enforcement.

Andrion et al. identified biological, chemical, and physical hazards in pathology, highlighting high tuberculosis risk with a six-fold increase among pathology workers in Japan and formaldehyde exposure at levels up to 8.0 ppm in certain pathology tasks​ [16]. Our study aligns with these concerns but focuses on quantifying occupational health issues in Indian pathologists, where 56.2% (N=82) reported neck pain and 66% (N=96) reported formalin intolerance. Unlike Andrion et al., who emphasized structural safety protocols, our findings stress the need for accessible ergonomic tools and safety practices tailored to resource-limited settings.

Another study by Sarwar et al. examined occupational hazards among Pakistani pathologists, finding a high prevalence of musculoskeletal issues (93.2%) and visual strain (90.6%), which closely aligns with our findings of 56.2% neck pain and 47.3% (N=69) back pain, though our musculoskeletal rates are slightly lower​ [17]. Both studies underscore the need for ergonomic interventions, with Sarwar et al. further highlighting significant psychological distress (90.1%)-a challenge noted in our study as well, albeit to a lesser extent. Their call for enhanced workplace design and regular ergonomic practices is highly consistent with our findings, reinforcing these areas as critical for well-being in pathology.

Similarly, Yahyaei et al. conducted a study in Iranian hospitals, which revealed that formaldehyde levels in pathology labs ranged from 0.0192 to 0.326 ppm. These levels often exceeded the National Institute for Occupational Safety and Health (NIOSH) limit (0.016 ppm) but were below the Occupational Safety and Health Administration (OSHA) threshold (0.75 ppm)​ [18]. In contrast, our study reported that 66% of respondents had adverse reactions to formalin exposure, emphasizing health impacts rather than precise exposure levels. Both studies underscore formaldehyde's health risks, but Yahyaei et al. highlight exposure monitoring, whereas our findings call for broader preventive practices and affordable safety measures.

Our study indicated a significant presence of chemical hazards as well. While Siow et al. focused on the neurological implications of solvent exposure, our findings highlighted musculoskeletal and respiratory impacts, with 56.2% of pathologists experiencing neck pain and 47.3% reporting back pain, illustrating a broader range of health risks within pathology work environments [19].

Implications of this study

The findings of this study underscore the urgent need for implementing comprehensive safety measures tailored to the specific occupational hazards faced by pathologists. Key recommendations include the mandatory use of ergonomic tools, such as adjustable chairs and microscopes designed to reduce musculoskeletal strain, and policies enforcing the regular use of cut-resistant gloves to prevent injuries during procedures. Establishing formal reporting mechanisms for injuries and chemical exposures is also critical, as these systems enable monitoring and timely intervention. Additionally, regular health screenings to detect early signs of occupational illnesses, such as chemical intolerance and respiratory issues, can mitigate long-term health impacts on pathologists. Also, pathologists with chronic conditions such as diabetes mellitus, hypertension, and other treated illnesses participated in the study. However, potential biases related to neck pain, low back pain, and refractive errors cannot be excluded.

Adoption of these safety measures is often hampered by barriers such as cost constraints, especially in resource-limited settings where high-quality ergonomic equipment is less accessible. Lack of awareness about the long-term benefits of ergonomic interventions and the perceived discomfort associated with protective gear also contribute to resistance among pathologists. To address these challenges, healthcare institutions should consider subsidizing essential ergonomic and protective tools, providing training on their correct use, and actively promoting a culture of workplace safety. Raising awareness about the risks of inaction and the health benefits of these measures could drive broader adoption and compliance.

Limitations of this study

While our study provides valuable insights into the occupational health challenges faced by pathologists, it is not without limitations. The use of an online questionnaire and printed forms may introduce selection bias, as only those willing and able to participate were included. This could skew the results, as individuals experiencing more severe occupational hazards may have been more likely to respond. Additionally, the self-reported nature of the data introduces the possibility of response bias, where participants may underreport or overreport certain health issues. The response coming from 146 out of 1000 participants, although diverse, is relatively small and limits the generalizability of the findings. Moreover, our study did not cover all the states and regions in India equally, and the results may not be entirely applicable to other regions or countries with different healthcare infrastructures and practices.

## Conclusions

This study sheds light on the significant occupational health challenges pathologists in India face, especially in terms of musculoskeletal disorders, needlestick and cut-related injuries, and formaldehyde exposure. While many pathologists are aware of the risks, the actual implementation of protective measures such as ergonomic tools and safety gear remains lacking. This gap, largely due to cost and accessibility issues, needs immediate attention. Institutional investment in ergonomic tools and mandatory safety training programs can help address such issues. 

Our findings highlight the urgent need for ergonomic interventions, safety protocols, and awareness campaigns targeting occupational health in pathology. Future research should explore the impact of region-specific challenges and assess the long-term efficacy of safety interventions. By prioritizing these changes, we can help reduce injury rates and create a healthier, safer work environment for pathologists, ensuring they can continue their critical work without compromising their own health.

## Appendices

Questionnaire

Informed consent form for participation in survey
